# Application Value of Evidence-Based Care in Patients with Lung Cancer Chemotherapy

**DOI:** 10.1155/2022/5747712

**Published:** 2022-07-30

**Authors:** Ying Chen, Hong Xu, Yun Cheng, Yuan Qian

**Affiliations:** ^1^Tumor Building, Affiliated Hospital of Jiangnan University, Wuxi City, 214061 Jiangsu Province, China; ^2^Tumor Building, Nursing Department, Affiliated Hospital of Jiangnan University, Wuxi City, 214061 Jiangsu Province, China

## Abstract

**Objective:**

The present research project is aimed at elucidating the application value of evidence-based care (EBC) in patients with lung cancer (LC) chemotherapy.

**Methods:**

Ninety-four advanced LC patients visited between March 2019 and February 2021 were retrospectively selected. Based on the type of care, 44 cases who used routine nursing were set as the control group (CG), and 50 patients who received EBC were included in the research group (RG). The pain degree, adverse mood, and individual fatigue of patients were assessed, using the Visual Analogue Scale (VAS), Self-Rating Anxiety/Depression Scale (SAS/SDS), and Cancer Fatigue Scale (CFS), respectively. Besides, patients were assessed for treatment compliance, self-efficacy, and life quality using the treatment compliance questionnaire, General Self-Efficacy Scale (GSES), and Quality of Life Questionnaire Core 30 (QLQ-C30), respectively.

**Results:**

The VAS, SAS, and SDS scores were lower in RG versus CG after nursing intervention. RG scored lower in the dimensions of physical, affective, and cognitive fatigue in terms of individual fatigue assessed by the CFS and higher in various domains of the QLQ-C30 score after nursing intervention. Besides, higher treatment compliance and self-efficacy were determined in RG as compared to CG.

**Conclusions:**

In addition to improving the treatment compliance, self-efficacy, and life quality of patients with LC chemotherapy, EBC can effectively alleviate their pain, adverse psychological mood, and individual fatigue, which deserves to be promoted in clinical application.

## 1. Introduction

Lung cancer (LC) is a fatal cancer represented by non-small-cell lung cancer (NSCLC), which causes approximately 2 million deaths worldwide every year [1]. The disease, originated from the bronchial epithelium or glands of the lungs, has the characteristics of high incidence and recurrence rate, with a five-year survival of merely 16.6% [2]. LC patients generally present with no obvious early symptoms, resulting in the fact that most of them are diagnosed in the middle and late stages with clinical presentations such as chest pain, hemoptysis, cough, and dyspnea [3]. Chemotherapy, a common treatment for patients with advanced LC, may also lead to adverse emotions such as irritability, depression, and cancer-related fatigue [4, 5], all of which will not only exert varying degrees of negative effects on the self-efficacy and life quality of LC patients undergoing chemotherapy but also reduce patients' treatment compliance that lowers their treatment compliance [6, 7]. This puts forward a demand for the management optimization of patients with LC chemotherapy, and exploring an effective and reliable high-quality nursing model is of positive significance for the rehabilitation of such patients [8].

Routine nursing intervention for LC patients undergoing chemotherapy often neglects psychological support, comfort care, pain threshold management, etc., which is difficult to mobilize patients' confidence to overcome the disease, resulting in a treatment outcome far from satisfactory [9]. Evidence-based care (EBC) is an intervention model that continuously improves nursing guidance and adjusts the practice process based on credible and scientific research results and past clinical experience [10]. Previous studies have shown that EBC has been recognized in different disease settings such as acute cerebral infarction, acute coronary syndrome, and postpartum depression, playing an active part in the treatment of patients, promoting patients' rehabilitation, and improving their treatment experience [11–13]. In addition, EBC has been applied clinically in LC patients receiving combined chemotherapy, which not only helps to reduce pain but also improves patients' quality of life and clinical satisfaction [14]. Nowadays, EBC has become a global nursing standard, which has the necessity and guiding advantages for healthcare systems, patients, and medical staff. However, its application in nursing practice is still relatively slow [15]. Therefore, in this study, we will compare the application value of EBC with conventional nursing in patients with LC chemotherapy, so as to verify its application advantages in such a medical background, and make a contribution to the clinical promotion of EBC and the management optimization of patients with LC chemotherapy.

## 2. Materials and Methods

### 2.1. General Case Data

This research was conducted after obtaining approval from the Affiliated Hospital of Jiangnan University Ethics Committee. Ninety-four advanced LC patients visited between March 2019 and February 2021 were retrospectively selected and grouped according to different nursing patterns, with 44 cases receiving conventional care included in the control group (CG) and 50 cases receiving EBC assigned to the research group (RG). CG included 24 males and 20 females, with an average age of 59.86 ± 8.37 years and a disease course of 4.66 ± 2.03 years, while RG was composed of 29 males and 21 females that averagely aged 60.18 ± 10.68 with a disease course of 4.84 ± 2.24 years. The two cohorts were comparable in gender, age, disease course, and other general data (*P* > 0.05). The subjects not only knew the research purpose but also signed and provided the informed consent form.

### 2.2. Eligibility Criteria

The following are the inclusion criteria: diagnosis of advanced LC, age ≥ 18, voluntary chemotherapy and regular treatment in our hospital, normal cognitive and communication skills, in line with the chemotherapy indications, and life expectancy > 6 months.

The following are the exclusion criteria: severe organ diseases, other malignant tumors, presence of mental illness or history of mental illness, and patients with limited mobility or otherwise unable to complete all methods of care. The patient selection flowchart can be seen in Figure 1.

### 2.3. Nursing Measures

CG received routine care. Patients were required to follow the doctor's instructions for appropriate treatment and care. During the treatment, the nursing staff paid close attention to patients' vital signs and made strict records and gave pain-relieving and targeted interventions to those with severe pain and complications. Meanwhile, the nurses distributed disease guidebooks to patients, patiently imparting their knowledge of health education and explaining precautions related to disease and treatment.

RG received EBC, the details of which are as follows:

1. Team building and scheme formulation: an EBC team composed of professional nurses and doctors was set up, and the team members were given professional training in EBC. Members of the team recorded patients' clinical data, reviewed relevant literature, and understood patients' nursing needs to develop reasonable nursing plans for them based on professional knowledge and disease analysis
2. Summary of nursing experience: according to previous medical records of LC patients undergoing chemotherapy, the possible complications, treatment methods, and corresponding causes of complications were summarized, and nursing experience was summed up to find potential solutions
3. Health education: health education related to disease and chemotherapy was given to patients, and the characteristics, symptoms, treatment, prognosis, and other knowledge related to LC were told to patients in an easy-to-understand language, so as to establish disease-related awareness for patients to cope with the disease more calmly. Prior to receiving chemotherapy, patients were popularized about chemotherapy drugs and frequency of use and other related information. Moreover, the medical staff patiently listened to and answered the questions raised by patients
4. Nursing of complications: according to the related risk factors and past pathology of patients with LC chemotherapy, preventive measures were taken to minimize the risk of complications
5. Psychological nursing: patients were given personalized psychological interventions taking their family, educational background, and disease development into consideration. Through strengthening communication, patients' emotions were appeased in time to reduce their psychological pressure. And by giving positive psychological hints and encouragement, patients were helped to build confidence in overcoming diseases and eliminate negative emotions and resistance to treatment as far as possible
6. Pain care: pain assessment was performed on all the enrolled patients. Besides, patients were briefed on pain and pharmacological remission and were told to follow the doctor's advice to take analgesics. The pain threshold of patients was also raised through distraction when they were in pain
7. Posture nursing: the medical staff gave patients guidance on postures and appropriately assisted patients to be in a comfortable position to avoid pressure ulcers
8. Exercise and diet care: patients were given scientific and appropriate exercise guidance based on their personal information and condition, so as to help them improve immunity and accelerate recovery. In addition, nurses gave corresponding dietary guidance to patients according to their eating habits and advised them to eat more high-protein foods and fruits
9. Discharge guidance: upon discharge, patients were instructed to take medicine scientifically and avoid increasing or decreasing the dosage or discontinuing the drugs by themselves. Besides, they were reminded that optimistic attitude, peaceful mood, and good living habits were the keys to stabilizing the condition and promoting rehabilitation. Patients were also told to see a doctor in time in case of any abnormalities

### 2.4. Endpoints

1. Degree of pain: the Visual Analogue Scale (VAS) [16], with a score of 0-10 and the score directly proportional to the pain degree, was used for pain assessment
2. Adverse mood: the Self-Rating Anxiety/Depression Scale (SAS/SDS) [17], both with a score ranging from 0 to 100 and the score directly proportional to negative emotions, were adopted for adverse mood evaluation
3. Individual fatigue: the Cancer Fatigue Scale (CFS) [18], which included three dimensions of physical (0-28 points), emotional (0-16 points), and cognitive fatigue (0-16 points), was employed for individual fatigue assessment. The score was positively related to the degree of fatigue
4. Treatment compliance: patients' treatment compliance was evaluated by the questionnaire of treatment compliance. Complete compliance was indicated if the patient was highly cooperative with the guidance of nurses and completed the guidance on time; basic cooperation with the guidance of nurses was regarded as partial compliance; failure to cooperate fully with the nursing staff and avoidance of nursing guidance is considered noncompliance
5. Self-efficacy: patients' self-efficacy was assessed by the General Self-Efficacy Scale (GSES) [19], a measurement with a score ranging from 0 to 145 and the score positively proportional to the level of self-efficacy
6. Life quality: the Quality of Life Questionnaire Core 30 (QLQ-C30) was used to evaluate patients' quality of life from five domains [20]: role, physical, social, cognitive, and emotional functioning. The score of each domain ranges from 0 to 100, and the score is proportional to the quality of life level

Among the above measures, the degree of pain, adverse mood, and individual fatigue were primary endpoints, while the others were secondary endpoints. In addition, all the above indicators were tested before and 6 months after nursing.

### 2.5. Statistics and Methods

GraphPad Prism 6 (GraphPad Software, San Diego, USA) was used for data analysis and image export. The counting data were represented as case/percentage (*n* (%)), and a chi-square test was employed for intergroup comparisons. Denoted by mean ± SD, the measurement data were compared by independent sample *t*-test between groups and by the paired *t*-test among different time periods. A significance level of *P* < 0.05 was used in all analyses.

## 3. Results

### 3.1. EBC Effectively Alleviates Pain of Patients with LC Chemotherapy

We compared and analyzed the pain levels of two groups of patients after nursing intervention by the VAS (Figure 2), in order to evaluate the impact of the two nursing methods on the relief of pain symptoms in patients with LC chemotherapy. The results showed no significant difference in VAS scores between groups prior to intervention (*P* > 0.05), while significant pain relief was observed in both cohorts after intervention (*P* < 0.01), with lower VAS scores in RG as compared to CG (*P* < 0.01).

### 3.2. EBC Significantly Mitigates Adverse Mood in LC Patients Undergoing Chemotherapy

SAS and SDS scores in both groups were recorded before and after nursing intervention (Figure 3). Similarly, the two scores were nonsignificantly different between groups prior to intervention (*P* > 0.05) and decreased notably in both cohorts after that (*P* < 0.01). The postintervention SAS and SDS scores were statistically lower in RG versus CG (*P* < 0.01).

### 3.3. EBC Significantly Reduces Individual Fatigue Degree and Improves Self-Efficacy of LC Patients Undergoing Chemotherapy

We evaluated patients' individual fatigue level and self-efficacy after nursing intervention by using CFS and GSES, respectively (Figure 4). The two scores differed insignificantly between groups before intervention (*P* > 0.05), while after intervention, the scores of physical, emotional, and cognitive fatigue in terms of individual fatigue assessed by the CFS were lower (*P* < 0.05) and the GSES score was higher in RG (*P* < 0.01), with statistical significance as compared to CG.

### 3.4. EBC Significantly Improves Treatment Compliance of Patients with LC Chemotherapy

Patients' compliance with treatment was evaluated through the compliance questionnaire (Table 1). RG using EBC was found with higher treatment compliance than CG treated with routine care (*P* < 0.05).

### 3.5. EBC Effectively Enhances Life Quality of Patients with LC Chemotherapy

The QLQ-C30 scores were measured before and after intervention to analyze the impact of the two models of care on patients' life quality (Figure 5). The data also determined no statistical difference in QLQ-C30 scores between groups prior to intervention (*P* > 0.05), while the score of each domain of the QLQ-C30 in RG after intervention was significantly higher than that before intervention and CG (*P* < 0.01).

## 4. Discussion

LC is one of the prime reasons for global cancer-related deaths, with most patients being not diagnosed at an early stage due to the presence of nonspecific clinical manifestations [21]. The common clinical treatments for patients with nonearly LC are radiotherapy and chemotherapy [22]. Although chemotherapy provides some benefits for LC patients, it may also lead to more serious complications that make patients overwhelmed [23], which will further affect their confidence to overcome the disease and cause certain psychological pressure, posing varying degrees of threat to patients' treatment compliance and self-efficacy [24]. We believe that providing high-quality EBC services to patients with LC chemotherapy will be more conducive to promoting their recovery, and we hereby report our findings.

LC patients will experience physiological pain caused by chemotherapy during the treatment process. In addition, chemotherapy will kill a large number of healthy cells while destroying cancer cells, which will lead to decreased immunity, organ dysfunction, nausea, vomiting, fatigue, hair loss, and other adverse events [25, 26]. In our study, both nursing methods played a certain role in relieving pain in patients with LC chemotherapy, but the VAS score of RG under EBC intervention was significantly lower compared with CG, suggesting that EBC has better pain-relieving effects than conventional nursing for such patients, consistent with the study of Liu et al. [14]. In the research of Zhang et al. [27], it is also pointed out that EBC is helpful to alleviate the eating pain of children with severe hand-foot-mouth disease. This is because under EBC intervention, medical staff will not only give pain assessment and analgesics but also conduct pain threshold and in vitro management of patients, all of which contributes to minimized pain degree in patients [28]. On the other hand, LC patients are prone to adverse mood after receiving chemotherapy, which is not only detrimental to the patient's recovery but also adversely affects treatment compliance, leading to an increased risk of relapse [29]. We observed lower SAS and SDS scores in RG after nursing compared with CG, indicating that EBC can significantly improve the adverse psychology of patients with LC chemotherapy, similar to the findings of Shen et al. [28]. EBC for LC patients undergoing chemotherapy also includes interventions for psychological disorders. Medical staff will provide personalized psychological interventions in combination with patients' personal information and do their best to help relieve patients' psychological stress and other adverse mood. In terms of individual fatigue and self-efficacy, RG exhibited lower CFS scores in the dimensions of physical, emotional, and cognitive fatigue than CG, as well as higher GSES scores, demonstrating that EBC is helpful to mitigate individual fatigue and enhance self-efficacy of LC patients undergoing chemotherapy. In addition, RG that received the EBC intervention also demonstrated higher treatment adherence. The above results are all consistent with those reported by Zhang et al. [30]. Under EBC, LC patients can gain a higher sense of self-esteem, because medical staff give patient responses, as well as disease-related cognition popularization, exercise, diet, and discharge guidance. Undoubtedly, professional support in all of the above aspects exerts positive effects on the alleviation of individual patient fatigue, and improvement self-efficacy, treatment compliance, and quality of life. Finally, through the QLQ-C30 scale, we also confirmed that the QLQ-C30 score of LC chemotherapy patients under EBC intervention improved more significantly in terms of role, physical, social, cognitive, and emotional functioning, better than the conventional nursing, suggesting that EBC was also significantly superior to conventional nursing in improving patients' quality of life.

Still, there are some limitations to be addressed in this study. First, the analysis of sleep quality and respiratory function of patients with LC chemotherapy should be supplemented to help further understand the potential advantages of EBC. Second, the sample size of the experimental subjects is small, and increasing the sample size will help to further improve the universality of research results. Finally, the evaluation indexes of pain degree, individual fatigue, treatment compliance, self-efficacy, and quality of life of LC patients undergoing chemotherapy are relatively single. The nursing strategy can be further optimized if we can supplement relevant analysis of influencing factors on the treatment compliance of patients with LC chemotherapy. Future studies will be gradually refined from the above angles. In addition, the contribution of this study to the subject area and its novelty is as follows: first, starting from the common negative states of LC patients undergoing chemotherapy, such as pain, adverse mood, and individual fatigue, it is confirmed that EBC has a significant inhibitory effect on the above aspects; that is, it can significantly reduce patients' pain, bad mood, and individual fatigue. Second, in terms of self-efficacy, treatment compliance, and quality of life, it is proved that EBC has a significant positive impact on the above aspects; namely, it can significantly enhance patients' self-efficacy and treatment compliance, contributing to improved life quality of such patients. The above provides a new theoretical basis for the nursing choice of patients with LC chemotherapy.

All in all, EBC is effective in the treatment of patients with LC chemotherapy, which can significantly reduce their pain and discomfort, relieve adverse mood and individual fatigue, and improve their treatment compliance, self-efficacy, and quality of life.

## Figures and Tables

**Figure 1:** Patient selection flowchart.

**Figure 2:** Pain levels of patients with lung cancer undergoing chemotherapy. The VAS score of the research group after nursing was significantly lower than that before nursing and the control group. Note: ^∗∗^*P* < 0.01. Independent sample *t*-test was used for data comparison between groups and paired *t*-test for data comparison before and after nursing.

**Figure 3:** SAS and SDS scores of patients with lung cancer undergoing chemotherapy. (a) The SAS score of the research group after nursing was lower than that before treatment and the control group. (b) The SDS score of the research group after nursing was lower than that before treatment and the control group. Note: ^∗∗^*P* < 0.01. Data comparison between groups and that before and after nursing were performed by independent sample *t*-test and paired *t*-test, respectively.

**Figure 4:** CFS and GSES scores of patients. (a) Physical fatigue scores of two groups of patients after nursing intervention. (b) Emotional fatigue scores of two groups of patients after nursing intervention. (c) Cognitive fatigue scores of two groups of patients after nursing intervention. (d) GSES scores of two groups of patients after nursing intervention. Note: ^∗^*P* < 0.05 and ^∗∗^*P* < 0.01. Data comparison between groups and that before and after nursing was performed by independent sample *t*-test and paired *t*-test, respectively.

**Figure 5:** Quality of life scores of lung cancer patients undergoing chemotherapy. (a) Role function scores of two groups of patients after intervention. (b) Physical function scores of two groups of patients after intervention. (c) Social function scores of two groups of patients after intervention. (d) Cognitive function scores of two groups of patients after intervention. (e) Emotional function scores of two groups of patients after intervention. Note: ^∗∗^*P* < 0.01. Data comparison between groups and that before and after nursing was performed by independent sample *t*-test and paired *t*-test, respectively.

**Table 1:** Treatment compliance of two groups (*n* (%)).

Groups	*n*	Complete compliance	Partial compliance	Noncompliance
CG	44	18 (40.91)	14 (31.82)	12 (27.27)
RG	50	28 (56.00)	18 (36.00)	4 (8.00)
*χ* ^2^ value	—	6.317		
*P* value	—	0.043		

Note: data differences between groups were analyzed by the chi-square test.

## Data Availability

The labeled datasets used to support the findings of this study are available from the corresponding author upon request.
